# Novel Antibacterial Resin-Based Filling Material Containing Nanoparticles for the Potential One-Step Treatment of Caries

**DOI:** 10.1155/2019/6367919

**Published:** 2019-03-13

**Authors:** Natalia Angel Villegas, M. Jazmin Silvero Compagnucci, Martin Sainz Ajá, Diamela María Rocca, María Cecilia Becerra, Gustavo Fabián Molina, Santiago Daniel Palma

**Affiliations:** ^1^Unidad de Investigación y Desarrollo en Tecnología Farmacéutica (UNITEFA), CONICET y Departamento de Ciencias Farmacéuticas, Facultad de Ciencias Químicas, Universidad Nacional de Córdoba, Ciudad Universitaria, X5000-Córdoba, Argentina; ^2^Instituto Multidisciplinario de Biología Vegetal (IMBIV), CONICET y Departamento de Ciencias Farmacéuticas, Facultad de Ciencias Químicas, Universidad Nacional de Córdoba, Ciudad Universitaria, X5000-Córdoba, Argentina; ^3^Departamento de Materiales Dentales, Facultad de Odontología, Universidad Nacional de Córdoba, Ciudad Universitaria, X5000-Córdoba, Argentina

## Abstract

The aim of this work was to study the application of resin filling containing nanomaterials for the potential treatment of caries. Zinc nanoparticles (ZnO@NP, 50 nm) were chosen for their antimicrobial capacity against aerobic bacteria, and here, they have proved to be bactericidal against anaerobic bacterial strains (*Streptococcus mutans*, *Streptococcus mitis*, and *Lactobacillus* spp.). Potential mechanism of action is proposed based on microbiological assays and seems to be independent of oxidative stress because the nanoparticles are effective in microaerophilic conditions. The loading of nanoparticles on the demineralized dental surface and their infiltration power were significantly improved when ZnO@NP were carried by the resin. Overall, this material seems to have a high potential to become a one-step treatment for caries lesions.

## 1. Introduction

Caries is a multifactorial disease characterized by the multitissue destruction in the tooth as a consequence of the demineralization caused by the acids generated by bacterial plaque. The bacteria produce these acids as a by-product of their metabolism of carbohydrates and then diffuse into dental hard tissues and dissolve their mineral contents leading to decalcification. Ultimately, this process usually results in the formation of a cavity in the tooth [1]. In this infectious disease, the enamel and dentin are also largely affected by demineralization due to the acids [2]. Caries is one of the most prevalent diseases in humans, and it remains a challenge to the medical and dental profession [3]. Despite the overall decline in caries prevalence in developed countries, this disease continues to be an important problem in the adult population of both developing and industrialized countries [4]. Nowadays, the treatment of caries (or root decay) consists of several phases, and therefore, patients tend to quit it before a full restoration is achieved. The first step in the “root canal treatment” (RCT) is the elimination of the infection, followed by filling of the cavity and reconstruction of the affected dental piece so that it recovers its functionality completely. Resin composites emerged as a good option for this last part due to their aesthetics and direct filling capabilities. However, they have one unsolved issue. The resin porous easily accumulates new bacterial plaque, leading to recurrent infections and, even worse, to more invasive treatment to remove it. Because caries at the restoration margins or surface is very often found, it would be highly desirable for the composite to have antibacterial and remineralization power [5]. Recent studies indicate that nanotechnology could provide novel strategies in the prevention and treatment of dental caries [6]. Several attempts have been made to modify the resins in order to provide antibacterial effects. In most of the experiments, antibacterial agents were incorporated into filling materials in order to inhibit the microbial attachment and dental plaque accumulation on their surfaces [7]. Moreover, nanomaterials have shown great potential for the inhibition of the demineralization process, remineralization of the dental structure, and the death of the pathogens involved in the caries lesion. This antibacterial effect is mainly attributed to the high surface area to volume ratio. In addition, the small size of these particles makes penetration through bacteria membranes easier resulting in higher antimicrobial activity [8]. Metal nanoparticles (i.e., silver and zinc) have gained significant interest over the years due to their remarkable antimicrobial properties. Silver nanoparticles are among the most used antibacterial agents incorporated into resin filler materials; however, the discoloration caused by the reduction of silver ions to metallic silver has been considered a major problem. Recently, new nanoantibacterial agents as zinc oxide nanoparticles (ZnO@NP), have been introduced, which theoretically will not cause discoloration, are nontoxic, and are biocompatible which make them suitable for use in humans [9, 10]. The aim of this work was to assess the effect of ZnO@NP incorporated into resin composite for the potential one-step treatment of caries lesion.

## 2. Experimental

### 2.1. Bacterial Strains

*Streptococcus mutans*, *Streptococcus mitis*, and *Lactobacillus* spp. were acquired from the Strain Collection of the Special Bacteriology Service (CCBE), INEI-ANLIS from Instituto Malbrán (Buenos Aires, Argentina).

These strains were always handled and kept in microaerophilic conditions using an anaerobic jar and were grown in thioglycollate broth with a colorimetric indicator or blood supplemented agar, according to the experiments needs.

### 2.2. Nanoparticles and Bacterial Media

Spherical ZnO@NP (CAS N° 1314-13-2) in the form of a white powder were purchased from Sigma Aldrich and used without modifications, size <50 nm. DMEM and brain-heart infusion were from Britania Lab.

Thioglycollate broth was also purchased from Britania Lab and freshly made and sterilized; also, it was heated in a mild water bath every time prior to use until its color indicates no oxygen dissolved in the liquid. Icon® resin was purchased from DMG Chemisch-Pharmazeutische Fabrik, Hamburg (composition based on methacrylate resin matrix, not fully disclosed by the manufacturer), and used straight from its syringe applicator. Blood-supplemented agar Petri dishes were purchase from Britania Lab.

### 2.3. Stability of ZnO@NP Suspensions

An equal amount of nanoparticles (2 mg/mL) was added to DMEM, brain-heart infusion, thioglycollate broth, and Icon® resin. Nanoparticles suspensions were kept at 37°C in a microaerophilic jar and were visually checked for aggregation or changes at *t* = 0, 2, 4, 6, 12, 24, 48, 72 h.

### 2.4. Antibacterial Activity

A large range between 0.2 to 2.2 mg/mL of ZnO@NP (in thioglycollate broth) was analyzed through the microdilution method (in a 96 well plate) against a bacterial initial inoculum (106 CFU/mL) freshly prepared (also in thioglycollate broth) from a single colony. All samples and controls (broth alone, ZnO@NP + broth, bacterial suspension alone) were conducted by triplicate, and the experiment was completely reproduced twice. The incubation of bacterial suspension with different nanoparticles concentration was made for 18 h at 37°C inside an anaerobic jar properly set for this purpose. After this period, 10 *μ*L aliquots of the samples with less and no turbidity (and controls) were dropped on blood agar Petri dishes to be incubated in the same conditions for 18 h. Finally, CFU counting was performed. Gram staining was done at the beginning and the end of the experiment to assure strains were not contaminated during the process.

### 2.5. ZnO@NP & Dental Surface Interaction Analysis

Completely developed third molars were obtained from the tooth bank for research proposes (Facultad de Odontología, Córdoba, Argentina—Faculty of Dentistry of the National University of Cordoba, Argentina—Ethical Committee Institutional doc N°3/2016). They were conserved in distilled water at 4°C and further processed for this study. 5 mm slices were cut from the Coronal Medium dentin region using a Buehler ISOMET Low-Speed Saw (origin: Alemania). The samples were polished with an abrasive disc and covered, except for a small window (3 × 3 mm) with purple nail polish as shown in Figure 1.

### 2.6. ZnO@NP Infiltration in Dental Samples

The aforementioned third molars slices, treated with ZnO@NP suspensions, were cut in half (90° to first cut). New slices were observed through SEM in order to discover the infiltration capacity of the nanomaterial carried in saline solution and Icon® resin.

### 2.7. SEM/EDS Analysis

Treated dental slices were treated with chromium for SEM/EDS observation (Lamarx Lab, Universidad Nacional de Córdoba, Argentina).

### 2.8. Statistical Analysis

All experiments were performed in triplicate, and numerical data are presented as means with error bars representing standard deviations.

## 3. Results and Discussion

Generally, bacteria are delimited by a cell membrane and cell wall. The outer border, the cell wall, is mainly constituted of peptidoglycan and is the one that keeps the osmotic pressure of the cytoplasm and the characteristic morphology [11]. The main difference between Gram-positive and Gram-negative bacteria is that the first ones have a multilayered membrane of peptidoglycan and the last ones have only one (of two) membranes composed of a thin peptidoglycan layer.

The overall exterior charge of both types of bacteria is negative; therefore, a better interaction is expected for positively charged drugs. The ZnO@NP employed in this study were chosen because they have an average size <50 nm (Figure 2) and a global positive zeta potential >35 mV. They are among the smallest and more stable one in acidic pH values, which is the media inside the mouth [12]. A good electrostatic interaction between bacteria and the selected nanoparticles is anticipated due to their global exterior charge. Particularly, this work assesses the effect of ZnO@NP on the caries producing anaerobic strains previously mentioned. All three of them are Gram-positive acid lactic producers. They produce a huge amount of this corrosive acid from food sugar. For all these reasons, evaluation of antibacterial agents must be done in sugar-rich acid bacteria culture media, with very low oxygen concentration. The ZnO@NP were more stable in thioglycollate broth than they were in brain-heart broth, so it was chosen to conduct the microbiology experiments. This could be because the last one has less concentration of salts that could promote nanoparticle aggregation. Great stability was also observed in DMEM and the resin (for interaction and infiltration tests). This could be due to the interaction of the ZnO@NP with acids groups from the media, which are known to act as stabilizers.[13].

Different methods have been adopted to investigate *in vitro* the antibacterial activity of nanoparticles although not all of them take into account the special requirements of these strains neither the nanomaterial properties [14]. For instance, the most frequently used one is the agar diffusion method, which is an indirect evaluation. In fact, there are multiple factors that determine the size of a zone of inhibition in this assay, including drug solubility, concentration in the disk and its diffusion rate through agar, and the thickness of the agar medium. Interpretation of the Kirby-Bauer disk diffusion assay provides only limited information on susceptibility and resistance to the drugs tested because all the abovementioned factors are not standardized. Even more important, the assay cannot distinguish between bacteriostatic and bactericidal activities. Kirby-Bauer disk diffusion methodology is not the right one to evaluate the antibacterial activity of ZnO@NP, considering the lack of solubility in water and low diffusion in agar. Other literature reports tell about how ZnO@NP conferred significantly decreased bacterial growth and proliferation [15, 16], which concurs with the experimental data of the present study. However, the turbidity method was usually applied alone, which it has its deficiencies as it examines both death and alive bacteria. In contrast, in the present study, measurements of bacterial suspensions' optical density (compared to controls with only nanoparticles suspension) were taken as an indication of growth inhibition; chosen samples were later seeded for further CFU counting. In this way, the MIC concentration for each strain was double checked, overcoming the disadvantages of individual methodologies.

The MIC of ZnO@NP was 1.2 mg/mL for *S. mitis* and as low as 0.6 mg/mL for *S. mutans* and *Lactobacillus*, but some effect could be observed at concentrations of just 0.2 mg/mL (Figure 3). These values are even lower than the ones depicted by Hojati et al. [17] probably because the several factors that influence the methodology they used, in fact, did not found any inhibition zone when doing agar diffusion but proved the effect of direct contact through.

The data presented here also support the antibacterial effect and provide an accurate value of the minimum inhibition concentration. Moreover, after checking the viability of the nanoparticles treated cultures by CFU counting, it can be assured that ZnO@NP are bactericidal for the tested strains. Importantly, the experimental setup allows demonstrating that they are bactericidal even in microaerophilic conditions, which are the actual conditions inside the caries cavity. One of the suggested antibacterial mechanisms for ZnO@NP is that they produce reactive oxygen species such as peroxide radical, which interfere in microbial growth. This could be true in an aerobic environment, but the results presented here show that this antimicrobial capacity is independent of the oxygen availability. Furthermore, there is no need to explore the photocatalytic activity of ZnO@NP, since they kill the anaerobic bacteria without any irradiation. This effect under dark has been observed by other researchers as well, but has never been tested in microaerophilic culture conditions [18, 19]. The antibacterial mechanism of ZnO@NP in dark is credited partially to the modification of the cell membrane activity after an electrostatic interaction [20]. At the same time, Zn^2+^ ions leaching in the growth media disrupt essential sugar metabolism and displace the magnesium ions which are essential for the bacterial enzyme systems [8]. All this combined could explain the effectiveness of this antibacterial agent.

Besides the antibacterial power, a potentially positive role on tissue regeneration is expected for ZnO@NP because Larsen and Auld [21] showed that zinc helps to stabilize proteins and has a protective effect when bonded to collagen regions that are sensitive to metal proteinase cleavage. They showed that zinc, forming zinc mono hydroxide, links catalytic ions to the lateral chain in the active site of carboxypeptidase A and inhibits it. Apparently, zinc acts as a matrix metalloproteinase (MMP) competitive inhibitor and decrease collagen degeneration in a single-bond hybrid layer and had no adverse effect on the bond strength [22]. Finally, SEM micrograph together with EDS measurements in treated dental slices (Figure 4) revealed that the loading of nanomaterial was 22 times higher (wt.%: 42.9 ± 1; Figure 4(c)) in dental samples treated with ZnO@NP carried in resin than in those treated with ZnO@NP at the same concentration in saline solution (wt.%: 1.9 ± 1; Figure 4(b)). The nanoparticles were measured by the quantitative EDS microanalysis in SEM, where the mass fractions or weight percents of the elements present in the sample are calculated. In contrast, no interaction at all was observed when the nanoparticles were suspended in water alone (Figure 4(a)). Interestingly, previous studies reported that the incorporation of nanoparticles into resin composites does not affect their adhesive properties but has indeed a positive effect on their mechanical characteristics. Alteration of resin properties is a common worry when adding nanoparticles, but ZnO@NP have no negative impact on the methacrylate material whatsoever. These nanoparticles conferred antimicrobial properties to the resin without altering the shear bond strength [2]. Another concern prior to clinical application is the toxicity level to human cells. Fortunately, they do not seem to be toxic at very low concentrations [1].

In addition to those benefits, ZnO@NP carried in resin showed better infiltration capacity than those in saline solution (Figure 5). As can be observed, Zn indicative of ZnO@NP could be found as deep as 1020 *μ*m from the dental surface when the methacrylate resin is used as a carrier. On the contrary, there is no Zn penetration when the nanoparticles are suspended in phosphate buffer saline (PBS). This ability to penetrate the dental sample is fundamental to reach deep bacterial infectious focuses.

## 4. Conclusions

With the evolution of caries lesion treatment shifting to “minimally invasive” techniques, restorative materials are endowed with increasing expectations for therapeutic effects. Current materials replace the missing volume of the tooth cavity although it would be useful for future restorative materials to not only replace the missing volume but also be bioactive and have beneficial therapeutic properties.

The nanotechnology is developing a new generation of bioactive therapeutic materials as an innovative concept for the development of materials with anticaries potential, capable of producing synergistic effects. Incorporation of nanoparticles into dental composites and adhesives proved to have multiple benefits: antibacterial capability and remineralization of tooth lesions. Although most of the studies on a new generation of antimicrobial, therapeutic, and bioactive resins are in vitro, in vivo studies are still needed. On the other hand, it is necessary to determine whether antibacterial resins induce bacterial drug resistance. Nonetheless, the new generation of antimicrobial resins, like the one proposed in this work, is expected to offer tremendous benefits to oral health. At the same time, these antimicrobial resins could establish the bases for other antimicrobial nanomaterials or filling. The results of this study are encouraging and open the doors to future multidisciplinary research and clinical studies that will allow the therapeutic value of nanotechnology-based restorative materials to be established.

## Figures and Tables

**Figure 1:** Experimental preparation of dental slices and ZnO@NP + resin treatment. That window was treated with a demineralizing solution (pH = 4.5, for 72 h with fresh solution every 24 h at 37°C) to produce the artificial caries lesion zone. Demineralizing solution composition: C_3_H_6_O_3_ (0.1 M), CaCl_2_ (3 mM), K_2_HPO_4_ (1.8 mM), carboxymethylcellulose 1%. Aliquots of ZnO@NP suspensions (1 mg/mL in H_2_O, saline 2 solution, and resin) large enough to cover the demineralized window were added dropwise and left to absorb for 5 minutes.

**Figure 2:** TEM images of ZnO@NP used for the experiments. Average size <50 nm. Scale bar: 100 nm.

**Figure 3:** Bacterial growth (Log CFU/mL) of *S. mutans* (blue), *S. mitis* (red), and *Lactobacillus* (green) treated with different concentrations of ZnO@NP in thioglycollate broth, during 18 h at 37°C, under microaerophilic conditions.

**Figure 4:** SEM/EDS micrographs of demineralized dental samples treated with ZnO@NP (in (a) H_2_O, (b) PBS, (c) Icon® resin).

**Figure 5:** Zinc (counts per second) vs depth (*μ*m), measured along the yellow line, of dental sample: treated with ZnO@NP + PBS (top right) and ZnO@NP + resin (bottom right). Illustrative SEM images of corresponding treated dental samples.

## Data Availability

Data generated or analyzed during this study are included in this published manuscript; however, more details are available from the authors upon reasonable request.

## Additional Points

*Future Perspective*. The treatment of caries lesion would have to evolve into some technique more practical and fast, that matches the requirements and standards of modern odontology including the concepts of minimally invasive restorative dentistry. Development of new materials, like the one presented here, is essential for this propose. For us, it is clear that in less than 10 years, one-step noninvasive treatment for caries would become routinary. In this framework, nanotechnology, and especially the use of metallic nanoparticles, will have a particular emphasis. *Executive Summary*. Caries lesion and current treatment: (i) caries is characterized by destruction in the tooth as a consequence of the demineralization caused by bacterial plaque; (ii) the routine treatment of caries consists of several phases which usually include the mechanical removal of dental tissue, and therefore, patients tend to quit it. Proposed nanomaterial: (i) the ZnO@NP used here have an average size <50 nm and a global positive zeta potential >35 mV; (ii) they are among the smallest and more stable ones in acidic pH values found inside the mouth; (iii) they have good electrostatic interaction with caries producing bacteria. Antibacterial activity: (i) the MIC of ZnO@NP was 1.2 mg/mL for *S. mitis* and as low as 0.6 mg/mL for *S. mutans* and *Lactobacillus*; (ii) in this case, antimicrobial activity was independent of oxygen availability. Interaction and infiltration of ZnO@NP with dental samples: (i) the load of nanomaterial on the dental surface was 22 times higher when ZnO@NP were carried in resin instead of PBS; (iv) a deep infiltration of ZnO@NP inside the molar sample could only be achieved when they were carried in the methacrylate resin.
